The article "Flux Dynamics in Y358 Superconductors" was retracted in 2012. Reasons: plagiarized text; overlap with other authors' work.

# Flux Dynamics in Y358 Superconductors

**DOI:** 10.3390/ma5050882

**Published:** 2012-05-18

**Authors:** Alireza Heidari, Seyedali Vedad, Niloofar Heidari, Mohammadali Ghorbani

**Affiliations:** Institute for Advanced Studies, Tehran 14456-63543, Iran; E-Mails: prof.alireza.heidari@instituteforadvancedstudies.us (A.H.); seyedali.vedad@yahoo.com (S.V.); heidarinilufar@yahoo.com (N.H.)

**Keywords:** high-T_c_ superconductor, thermally activated flux motion, transition temperature

## Abstract

Thermally activated flux motion and specific electric resistance in Y358 were studied under different magnetic fields ranging from 0 to 15 kOe. Through investigating the broadening of normal-superconducting transition, we found that the thermally-activated-flux-motion model can describe the electronic effect near the superconducting transition temperature. By modifying this model, specific electric resistance at different magnetic fields was calculated.

## 1. Introduction

Wu *et al*. [1] discovered a new compound, YBa_2_Cu_3_O_7_ or Y123, of the YBCO family with T_c_ = 92 K—above the liquid-nitrogen temperature—which was composed of copper-oxide layers. A year later, Y124 and Y247, with respective transition temperatures of 80 and 40 K, were discovered [2,3]. Y358 (Y_3_Ba_5_Cu_8_O_18_) has been recently synthesized, with a transition temperature of about 2 K higher than that of Y123 [4,5]. This compound consists of five CuO_2_ layers and three CuO chains in the unit cell.

Various models have been devised to analyze the broadening of electric-resistance transition region below the transition temperature of high-T_c_ superconductors under different magnetic fields. The flux-creep model, flux-flow model, and the model of phase slip, which results from fluctuations in superconductor order parameters, are being utilized to explain the broadening of specific-resistance transition in high-T_c_ superconductors under a magnetic field. In some high-T_c_ superconductors, a good fit has been observed by employing the Ambegaokar-Halperin (AH) model [6]. In some reports [7], a slight deviation from the AH model near T_c_ (ρ = 0) has been observed. The thermally-activated flux-creep (TAFC) model is more appropriate for studying this region. Here, we studied the magnetic properties and flux dynamics in Y358 through a TAFC model.

## 2. Experimental Section

The Y_3_Ba_5_Cu_8_O_18_ sample was synthesized through a standard solid-state technique. Stoichiometric ratios of the powders of CuO, BaCO_3_, and Y_2_O_3_ were mixed on a magnetic mixer, ground, calcined at 840 °C in air for 12 h, and cooled to room temperature for 5 h. The product was recalcined, reground, pressed under 10 ton/cm^2^, and sintered at 920 °C. The sample was synthesized at 890–930 °C in an oxygen atmosphere for 24 h. Afterwards, it was cooled to 500 °C, maintained in oxygen flow for 10 h, and then furnace cooled to room temperature [4,8]. Then, this sample’s electric resistance was measured using a four-probe method under different constant magnetic fields (H = 1, 2, 5, 8, 10, 12, and 15 kOe) perpendicular to the sample surface and electric current. The electrical joints were attached by silver glue. The broadening in the below-T_c_ region under different magnetic fields was investigated using a modified TAFC model.

## 3. Results and Discussion

Figure 1 shows the specific electric resistance of Y358 as a function of temperature under different magnetic fields ranging from 0–15 kOe. As can be observed, the applied magnetic fields slightly affect the normal-state electric resistance and only change the below-T_c_ transition region. The application of magnetic field broadens the transition region and reduces T_c_ (ρ = 0). For H = 15 kOe, T_c_ (ρ = 0) was observed to be 58 K. The broadening of specific-electric-resistance transition suggests that the sample is sensitive to the external magnetic field through dissipation phenomenon, which is caused by flow around fluids [9]. Such behavior is attributed to pinning energy. According to the TAFC model, the following equation defines the correlation between specific electric resistance and pinning energy [10,11,12,13,14]:

(1) $$\rho (H,T)=\rho_{0}\exp(-U(H)/k_{B}T)$$

where *ρ*_0_ denotes normal-state electric resistance. Assuming that the thermal activation process is performed, the pinning energy (*U*) corresponds to the slope of the lnρ-1/T curve at low temperatures. Figure 2 shows this curve plotted for Y358 at different magnetic fields.

**Figure 1:** Specific electric resistance of Y358 with respect to temperature under different magnetic fields ranging from 0–15 kOe.

**Figure 2:** The lnρ-1/T diagram of Y358 under different magnetic fields ranging from 0–15 kOe.

U/k_B_ and ρ_0_ are respectively obtained from the tail-end slope and intercept of these curves. The near-T_c_ (ρ = 0) region in most plotted curves does not show a good fit to a line. The values of ρ_0_ obtained through fitting the approximately linear parts of lnρ-1/T curves vary from 10^9^ to 10^21^ mΩ-cm, which is far larger than the normal-state electric resistance of Y358. Because electric resistance must equal ρ_0_ and roughly equal the normal-state resistance of transition onset when pinning energy is negligible, we should also consider the correlation between the activation energy and temperature [10]:

(2) $$U=U(H){\left(1-\frac{T}{T_{c}}\right)}^{\alpha }$$

where the value of *α* has been reported as 1, 1.5, and 2 for high-T_c_ superconductors [5,11,12]. We plotted the ln(ρ) − 1/T(1 − T/T_c_)^α^ curves for α = 1, 1.5, 2, 2.5, and 3 under a 2 kOe magnetic field (Figure 3a) to investigate the correlation between U and temperature and to find the appropriate value of α. Figure 3b shows these curves’ roughly linear region with line fitting. The value of R^2^ (fitting percentage) for α = 1, 1.5, 2, 2.5, and 3 was calculated as 0.96, 0.97, 0.99, 0.994, and 0.996, respectively (Figure 3b). The results of line fitting demonstrated that α = 3 shows a more appropriate fit to the curves. Also, the slight difference between α = 2 and 3 suggests that the system we studied is two-dimensional [15,16].

**Figure 3:** (**a**) The curves of lnρ *versus* 1/T(1 − T/T_c_)^α^ for α = 1, 1.5, 2, 2.5, 3 under a 2 kOe magnetic field; (**b**) The roughly linear parts of the curves in (a) with line fitting.

The ln(ρ) − 1/T(1 − T/T_c_)^2^ curves of Y358 under different magnetic fields are illustrated in Figure 4. As is evident, the slope of the curves, which determines the value of pinning energy, declines with amplifying magnetic field; consequently, pinning energy falls. Flux creep and crossing the potential barrier due to pinning centers are more easily performed and a reduction in potential barrier decreases the value of activation energy. At low temperatures, we fitted these curves’ roughly linear part with a line and report their slope and intercept in Figure 5. The slope of these curves’ tail end is equal to the value obtained for U(H).

**Figure 4:** The curves of lnρ *versus* 1/T(1 − T/T_c_)^2^ under different magnetic fields ranging from 0–15 kOe.

**Figure 5:** The linear fits of ln(ρ) − 1/T(1 − T/Tc)^2^ curves under different magnetic fields ranging from 0–15 kOe.

Figure 6 shows the effect of the applied magnetic field on the pinning energy U(H) for Y358. As can be seen, with amplifying magnetic field from 0 to 15 kOe, the rate of decline in pinning energy decreases and behaves exponentially. Under magnetic fields below 1 kOe, the pinning energy depends heavily on the value of magnetic field. This case should be investigated in the future.

**Figure 6:** The effect of the applied magnetic field on pinning energy.

## 4. Conclusions

By modifying the TAFC model and considering the temperature dependence of pinning energy, we observed the best linear fit for α = 3 at near-T_c_ temperatures, which demonstrates that Y358 is two-dimensional. Also, we found that pinning energy behaves exponentially with changing magnetic field. For the magnetic fields below 1 kOe, pinning energy is dramatically reduced with amplifying magnetic field; however for larger magnetic fields, pinning energy slightly declines with increasing magnetic field.

Application of a magnetic field reduces the intragranular T_c_^onset^ in Y358. However, it further affects the intergranular T_c_. The investigation of this phenomenon is one of the topics of our future studies.
